# The Expanding Universe of Prion Diseases

**DOI:** 10.1371/journal.ppat.0020026

**Published:** 2006-03-31

**Authors:** Joel C Watts, Aru Balachandran, David Westaway

## Abstract

Prions cause fatal and transmissible neurodegenerative disease. These etiological infectious agents are formed in greater part from a misfolded cell-surface protein called PrP^C^. Several mammalian species are affected by the diseases, and in the case of “mad cow disease” (BSE) the agent has a tropism for humans, with negative consequences for agribusiness and public health. Unfortunately, the known universe of prion diseases is expanding. At least four novel prion diseases—including human diseases variant Creutzfeldt-Jakob disease (vCJD) and sporadic fatal insomnia (sFI), bovine amyloidotic spongiform encephalopathy (BASE), and Nor98 of sheep—have been identified in the last ten years, and chronic wasting disease (CWD) of North American deer *(Odocoileus Specis)* and Rocky Mountain elk *(Cervus elaphus nelsoni)* is undergoing a dramatic spread across North America. While amplification (BSE) and dissemination (CWD, commercial sourcing of cervids from the wild and movement of farmed elk) can be attributed to human activity, the origins of emergent prion diseases cannot always be laid at the door of humankind. Instead, the continued appearance of new outbreaks in the form of “sporadic” disease may be an inevitable outcome in a situation where the replicating pathogen is host-encoded.

## Prion Diseases and Prion Proteins

Prion diseases, sometimes referred to as transmissible spongiform encephalopathies (TSE), affect a variety of mammals. These neurodegenerative diseases are incurable, with pathogenesis in the central nervous system leading slowly but inexorably to death. These diseases are exemplified in humans by Creutzfeldt-Jakob disease (CJD), while in cattle the head-line grabbing “mad cow” disease, bovine spongiform encephalopathy (BSE), immediately comes to mind. A remarkable feature of this class of diseases is the extended period of time between exposure to the infectious agent and manifestation of clinical symptoms. This period may typically be reckoned in decades for the syndromes in humans, but can be as short as 1.5 years in the case of iatrogenic disease [1]. In laboratory rodent models this period is usually less than one year. Although once attributed to hypothetical unconventional viruses, evidence has accumulated that these pathogens involve a fundamentally different type of replicative process—epigenetic templated protein misfolding—a process with some similarity to pathogenic events in several other (albeit nontransmissible) neurodegenerative diseases such as Parkinson disease and Alzheimer disease.

The infectious agent in prion diseases is believed to be composed of a single protein and, not surprisingly, this is dubbed the prion protein (PrP). The prion hypothesis states that a disease-associated and improperly folded form of PrP (generally termed PrP^Sc^) is derived from a benign membrane-displayed precursor protein, PrP^C^, encoded on Chromosome 2 and Chromosome 20 in mice and humans, respectively [2]. The epidemiological appearance of certain human prion diseases in genetic and sporadic forms (not the case with other classes of infectious pathogens) is also compatible with the concept of aberrant metabolism of a “host” cellular component. Indeed, a tri-modal epidemiological manifestation is a unique feature of prion diseases and unique in the realm of medical biology, blurring the dividing lines between metabolic and infectious diseases. In the case of inherited prion diseases such as familial CJD (now referred to as genetic CJD), vertical transmission is not by an infectious route but by germ-line inheritance of a mutated form of the prion protein. Here the mutations may lead to misfolding by encouraging the overrepresentation of transient folding intermediates [3]. Several examples are now known, and these have been reviewed elsewhere [4]. Sporadic prion disease is arguably the most fascinating and unpredictable epidemiological manifestation of all, and the curious mechanisms by which this might arise are discussed later. The best-documented sporadic disease is sporadic CJD (sCJD). This comes in several subvarieties, and it is known that a common asymptomatic polymorphism in the human *PRNP* coding region, either a methionine or a valine at codon 129, has a profound effect upon the appearance of this disease (an important modulatory role of this polymorphism is also apparent for genetic prion diseases such as genetic CJD (gCJD)). With regard to infectious disease manifestation, BSE is the best-known example. In this disease, infectivity is acquired by an oral route of administration. Exposure to BSE prions in Europe has lead to about 170 cases of variant CJD (vCJD) thus far.

## From PrP^C^ to PrP^Sc^

PrP^C^ is synthesized in the secretory pathway, and the mature form of mouse PrP^C^ is a 210 amino acid protein, N-glycosylated, and anchored to the cell surface by means of a glycosylphosphatidylinositol anchor. The structure of PrP^C^ consists of two domains: an N-terminal flexibly disordered domain which is capable of binding copper, and a C-terminal α-helical domain [5,6]. In contrast, PrP^Sc^ is enriched in β-sheet content and is characterized by its poor solubility in nondenaturing detergents, propensity for aggregation, and partial resistance to proteinase K (PK) digestion [7] (Figure 1). Digestion of PrP^Sc^ with PK results in an N-terminally truncated fragment originally called PrP27–30 in the case of scrapie infections and more generally termed PrP^res^, to denote protease-resistance in vitro. Although PrP^Sc^ appears to be more thermodynamically stable than PrP^C^, folding of N-terminally truncated recombinant PrP^C^ to the α-helical conformation takes place with rapid kinetics at neutral pH [8]. Since a substantial energy barrier exists between α-helical PrP^C^ and isoforms rich in β-structures [9], the resulting “kinetic trap” for nascent PrP^C^ synthesized at neutral pH overwhelmingly favors formation of the α-helical conformation, perhaps consistent with the observation that spontaneous formation of PrP^Sc^ (e.g., de novo genesis of sporadic disease such as sCJD, as discussed below) is not favored under physiological conditions. Although there is debate as to whether other proteins or accessory molecules participate in the refolding event in vivo [10–12], PrP^C^ is absolutely required for the disease process insofar as PrP knockout mice fail to develop disease when inoculated with prions [13].

**Figure 1:** Formation of PrP^Sc^ and Pathways to Disease (A–C) Structures of PrP^C^ and PrP^Sc^. (A) NMR structure of PrP^C^ with a notional addition of the N-terminal region (which is unstructured in NMR analyses). Copper ions (turquoise spheres) and coordinating side chains (dark blue) are shown. Note that the C-terminal globular domain has two short beta strands (turquoise arrows) and three α-helices (red; image courtesy of Glenn Millhauser, University of California Santa Cruz). (B) A structure for PrP^Sc^ deduced from electron microscopic analyses of purified material. The background represents the two-dimensional crystals of PrP27–30 after image processing and the foreground a notional structure for PrP^Sc^ with the central region of the protein rearranged into triangular stacked β-helices (image courtesy of Cedric Govaerts and Holger Wille, University of California San Francisco). (C) Linear representation of PrP^C^ and PrP^Sc^, and N-terminal truncation of PrP^Sc^ by proteinase K, to create PrP27–30. For illustrative purposes the conformational change in the centre of the molecule is shown by an altered color for helix A. Also note that other conformational changes may occur C-terminal to this position, but have been omitted for the sake of clarity. (D) Pathways to disease. In prion infections, conversion of PrP^C^ to PrP^Sc^ is initiated by a pre-existing seed of PrP^Sc^. In genetic diseases the mutant form of PrP^C^ denoted PrP^M^ may misfold and aggregate, and in some case acquire PrP^Sc^-like properties sufficient to initiate disease in inoculated recipient animals. In sporadic disease the mechanism of spontaneous misfolding to PrP^Sc^ is unknown.

## Prion Strains and Host Range

As replicating pathogens, prions do have two attributes that seem “viral-like.” The first is that they can exist in strains, that is to say, isolates appear to have distinctive phenotypic attributes within the same genotype of host (typically a mouse inbred strain). These attributes may include incubation time from inoculation to disease onset, neuropathology, the degree of N-glycosylation of PrP^Sc^, and the degree of resistance to proteinase K digestion in vitro. In a molecular sense, prion strains are thought to correspond to conformational subvarieties of PrP^Sc^ that are capable of accurately templating this three-dimensional information to nascent PrP^Sc^ molecules [14–17].

Prions are also like viruses in that they have host-range phenomena. They can adapt to certain host species and conversely, may falter (or at least be impeded) when introduced into a different species [18,19]. In an experimental setting two variables may be important for abrogating species barriers to “foreign” prions. The first is to match the primary sequence of the host PrP^C^ to the primary sequence of the PrP^Sc^ polypeptides in the inoculum of interest, first done for hamster prions by transgenetic means [20,21]. A second operational variable is to remove an interfering effect of the endogenous (typically mouse) PrP^C^ allele upon assay of heterologous prions, and this is accomplished by using a gene-ablated (*Prnp* ^0/0^) genetic background for the prion-inoculated animals [13,22]. These parameters still cannot be the whole story, though, as evidenced by the case of the bank vole, which—in spite of having PrP with seemingly unremarkable primary structure—is susceptible to prions from a number of mammals [23].

Overall, there is a distinctly biophysical flavor to prion replication that has no precise equivalent in the events that might typically preoccupy mammalian virologists, namely synthesis of the genome-length nucleic acids, synthesis of viral proteins required for propagation, and virion interactions with cell-surface receptors. Also, as may be appreciated, the distinction between “non-host” extrinsic chemistry and intrinsic physiological events is more slender in prion disease than for viral infections: in the latter case the infectious particle may be composed of many varieties of macromolecules and the molecular weight may rank in the millions. The proximity of prion protein misfolding and replication to normal cellular events can present unique challenges for diagnosis, and current procedures warrant description before tackling the mysteries of prion biogenesis and emerging diseases.

## Prion Gazing

### 

#### Static diagnostics.

Several techniques are used for postmortem diagnosis of prion disease [24] (Table 1). Brains of infected individuals usually exhibit pronounced spongiform change (areas of vacuolation), neuronal degeneration and death, astrogliosis, and occasionally, the accumulation of amyloid plaques containing aberrant PrP. Spongiform change can be observed using standard histological procedures, and abnormal PrP deposits can be viewed following pretreatment with formic acid and hydrated or hydrolytic autoclaving [25], to reduce the immunoreactivity of PrP^C^, prior to staining with a PrP-specific antibody (see Figure 2). Other diagnostic tests rely on the detection of PrP^res^ as a surrogate marker for PrP^Sc^. Following PK treatment, PrP^res^ can be detected using either a Western blot or an ELISA, with these strategies forming the basis for two of the most widely used commercial tests for BSE (from Prionics, Schlieren, Switzerland, and BioRad, Hercules, California, United States, respectively). A distinct approach, one that circumvents protease digestion, is the conformation-dependent immunoassay [16,26,27]. This method takes advantage of the differential availability of sequestered antibody epitopes between PrP^C^ and PrP^Sc^. An antibody is used which recognizes a central epitope with differential accessibility between PrP^C^ (available) and PrP^Sc^ (not accessible until thermal or chemical denaturation). Ratios are calculated between signals obtained by ELISA for the native and denatured forms of the test samples, which are then used to ascertain the presence of PrP^Sc^. In this technique there is the potential to detect soluble forms of PrP^Sc^ which may outnumber their insoluble and more protease-resistant counterparts. Lastly, antibodies have now been described which may react with determinants unique to PrP^Sc^ [28–31].

**Table 1:** Commonly Used Methods for Detecting TSE and PrP^Sc^

**Figure 2:** Pathology in CWD-Infected Animals (A) Histologic lesions of CWD in the dorsal motor nuclei of the vagus nerve within the medulla oblongata of a CWD-affected elk. Note spongiform change, intraneuronal vacuoles, and mild gliosis (hematoxylin and eosin stain, 100× magnification). (B) PrP amyloid deposit stained by immunohistochemistry (brown) and surrounded by vacuoles (original magnification 180×). (C)**** Perineuronal and extracellular deposits of abnormal PrP (PrP^CWD^, analogous to PrP^Sc^) in a CWD-affected mule deer (original magnification180×). (D) PrP^CWD^ deposits in the germinal centres of lymphoid follicles in the tonsils of a mule deer (immunohistochemistry, original magnification 50×).

#### Active diagnostics.

In contrast to static diagnostics which biochemically detect aberrant PrP, active diagnostics amplify PrP^Sc^ or infectivity in vivo or in vitro before a detection step or biological readout. The prion bioassay in mice is the most commonly used method for assaying infectivity in vivo. Following intracerebral inoculation of the test sample, mice typically succumb to prion disease following an incubation period of approximately 150 days (which is dependent on the strain of mouse and prion strain utilized). Although considered to be the gold standard, this bioassay system has a number of important drawbacks. Firstly, bioassays are expensive, labour intensive, and time-consuming. Second, unless mouse or rodent-adapted prions are being tested, these bioassays may be subject to species–barrier effects leading to prolonged incubation times or inefficient transmission of disease. Attempts to circumvent the species barrier have resulted in the development of transgenic indicator mice, mice which express PrP^C^ of the same amino acid sequence as the PrP^Sc^ in the test inoculum [12,32–35]. As mentioned, wild-type bank voles have an unexpected susceptibility to prion disease and these may prove versatile as a miner's canary for emergent diseases of unknown tropism.

Although invaluable, mouse bioassays are not high throughput. Another active technique, which is ten times faster than conventional bioassays and approximately two orders of magnitude cheaper, is the scrapie cell assay [36]. This cell culture-based method utilizes sublines of mouse N2a neuroblastoma cells that have been selected for enriched susceptibility to prions and measures the ability of a test sample to generate PrP^Sc^-positive cells. Following exposure, cells are split three times (to remove any PrP^Sc^ left over from the test sample), filtered onto the membrane of an enzyme-linked immunospot (ELISPOT) plate, digested with PK, and immunostained for PrP. Quantitation is performed using an ELISPOT system (a stereo microscope equipped with a camera and scanner linked to specialized software) and comparison to standard curves generated from titred samples results in a measure of the infectivity of the test sample. Greater sensitivity can be obtained if the scrapie cell assay is performed in endpoint titration format. One drawback of this technique is that attempts to use mouse-adapted prions other than the Rocky Mountain Lab isolate (such as the murine Me7 and 22A isolates) were unsuccessful [36].

A third active diagnostic technique, denoted PMCA (protein misfolding cyclic amplification), was developed by Soto and co-workers as a means of producing large quantities of PrP^res^ in vitro [37] (Figure 3). The method is loosely similar in a conceptual sense to nucleic acid PCR. Fresh brain homogenate from non-infected animals is used as a source of PrP^C^, and brain homogenate from scrapie-infected animals as a source of PrP^Sc^ [38]. In this analogy, PrP^Sc^ is akin to the rare nucleic acid target sequence of PCR, and PrP^C^ is akin to the cocktail of oligonucleotide primers and mononucleotides that allow de novo nucleic acid synthesis. Small amounts of infected material are diluted into normal brain homogenate and in vitro conversion—presumably a form of templated protein refolding—is allowed to proceed at 37 °C. A key ingredient is a subsequent sonication step, formally analogous to thermal denaturation of complementary DNA strands in a PCR reaction. Here, mechanical energy is used to break up newly formed PrP aggregates into smaller structures, with the latter providing new seeds for PrP^res^ formation in reiterations of the two-step procedure. In this way repeated cycles of conversion and sonication are performed in order to amplify any PrP^Sc^ present in the starting sample. Conversely, only modest amounts of PrP^res^ are generated if the sonication step is omitted [37,39,40].

**Figure 3:** Schematic Representation of the PMCA Procedure Brain homogenate from an infected animal (containing PrP^Sc^) is diluted into homogenate from a healthy animal (containing PrP^C^) and incubated at 37 °C. During this stage, some molecules of PrP^C^ are converted to PrP^res^ and are added to the growing PrP^res^ unit. Sonication breaks up PrP^res^ into smaller units, generating new seeds for conversion. These steps are repeated in a cyclic fashion in order to amplify the amount of PrP^res^ present in the initial sample. The stoichiometry and directionality of amplification depicted are for illustrative purposes only and are not meant to represent intrinsic properties of the system.

## The Expanding Universe of Prion Diseases

### 

#### vCJD and “mock sCJD” in humans.

Suitably equipped with diagnostic savvy we may now move to emergent prion diseases (Table 2). Here they have been classified either as diseases defined in the last ten years, or as diseases that have undergone a dramatic increase within the same time period. The first example, vCJD, was first recognized in 1996, and the occurrence of this disease as a consequence of the UK BSE epidemic has been described in detail elsewhere [41,42]. While large-scale screening programs of diverse livestock and cervid species prompted in greater part by the vCJD epidemic have increased the spectrum of prion diseases, surprises have also emerged in the context of the human disease. All clinically confirmed cases of vCJD have been of the codon 129 *M/M* genotype, and the one “case” of vCJD that has been sighted in a non-*M/M* genotype occurred in the form of an asymptomatic *M/V* heterozygote patient who received a blood transfusion from a vCJD donor [43]. This suggests that infections are proceeding at a slower pace in *M/V* and *V/V* individuals in the UK exposed to BSE prions, and that these individuals currently have subclinical disease. In agreement with these ideas, transgenic mice expressing just the human 129V form of PrP^C^ exhibit a significant barrier to infection with either BSE or vCJD prions, and those that do become infected have distinct neuropathological characteristics and propagate a different type of PrP^Sc^ from vCJD [44]. As expected, the majority of mice expressing human 129M PrP^C^ display the hallmarks of vCJD upon inoculation with BSE or vCJD prions, with one remarkable exception. A single mouse inoculated with BSE prions developed a disease indistinguishable from human sporadic CJD [33]. This result has led to the suggestion that a sliver of sCJD cases in Europe may have resulted from BSE exposure (i.e., are vCJD cases masquerading as sCJD), but since the “mock” sCJD resulting from oral exposure to BSE prions has the hallmarks of conventional sCJD type, establishing this inference will be tricky. In Switzerland, a country with documented cases of BSE, the incidence of sCJD underwent a 2-fold increase in 2001 [45]. However, a large-scale epidemiological study failed to find any changes in the characteristics of sCJD in the UK [46].

**Table 2:** Emerging Prion Diseases in Animals and in Humans

**Figure 4:** CWD in North America Geographical distribution in North America (A), and in expanded view of Alberta and Saskatchewan (B). Data in (A) is correct as of February, 2006, and reproduced with kind permission of the CWD Alliance. In (A), states or provinces where CWD has been diagnosed in captive populations are cross-hatched. CWD diagnosis in free-ranging animals is indicated by red circles. In (B), CWD diagnosis in free-ranging animals is indicated by red circles and in farmed animals with green circles. (C) Mule deer with clinical CWD showing emaciation and loss of body condition (photo courtesy of T. R. Spraker). (D) Elk with clinical CWD showing emaciation and excessive salivation (photo courtesy of E. S. Williams).

#### sFI in humans.

Whereas fatal familial insomnia is a genetic disease caused by a *PRNP D178N* mutation in *cis* to a methionine polymorphism at codon 129, more recent work has described a sporadic version of the same syndrome. To date, eight cases of sporadic fatal insomnia (sFI) have been reported [47–50], all of which resemble typical fatal familial insomnia and are homozygous for the methionine codon 129 polymorphism but lack any mutation in the *PRNP* gene. sFI has successfully been transmitted to mice and the resulting neuropathology and electrophoretic signature of PrP^Sc^ are indistinguishable from those obtained with mice inoculated with fatal familial insomnia isolates.

#### BASE in cattle.

Here, abnormal presentation of prion disease in two cattle in Italy was sufficiently distinct from BSE as to suggest a distinct neurological syndrome denoted bovine amyloidotic spongiform encephalopathy (BASE) [51]. Notable amongst the histopathogical features were deposition of amyloid plaques in the thalamus, subcortical white matter, and the olfactory bulb, while PrP^Sc^ detected by Western blotting did not have the preponderance of di-glycosylated PrP forms typical of BSE. Instead, the signature from this kind of analysis was most akin to that of type M/V2 sCJD (a subtype of sCJD characterized by Kuru-like plaques and so-called type 2 PrP^Sc^). Perhaps this may be related to observation that upon inoculation of “humanized” mice with BSE prions, a small group of mice propagated a prion with similarities to sCJD (see above) [33]. Results from BASE serial transmission experiments (to prove that BASE results from an infectious TSE agent) have not yet been published.

#### Nor98 in sheep.

A fourth emergent disease, sometimes referred to as atypical scrapie, was first detected in Norwegian sheep eight years ago [52]. There was no evidence of lateral or horizontal transmission, with cases (one per flock) observed in geographically dispersed locations. Furthermore, the novelty of this disease extended beyond these epidemiological observations to include distinctive genetic, biochemical, and histopathological signatures. These correspond to occurrence in supposedly scrapie-resistant ovine *Prnp* genotypes [53,54], protease resistant PrP of an unusually short type (~12 kDa) [52], and immunohistochemical detection of PrP^Sc^ deposition in the cerebellar cortex yet no obvious deposition in the medulla oblongata, which is the primary and earliest site of detection in classical scrapie. Thus far, PrP^Sc^ has not been found in the lymphoreticular system. Subsequent analyses have identified Nor98-like TSE cases in other countries, including France, Germany, Sweden, Portugal, and Belgium [53,55–57].

From the foregoing data, it is unclear whether labeling Nor98 as a type of scrapie is accurate, or is more of a reflexive action made on the basis of the host species. Irrespective of the wisdom of this label, a further twist in the story is that Nor98 has now been shown to be transmissible. Transmission of either Nor98 (Norwegian isolate) or discordant (atypical) scrapie cases (French isolates) to ovinized mice expressing the PrP^VRQ^ allele faithfully recapitulated the disease seen in sheep, highlighted by the presence of the ~12-kDa PrP^res^ band and the lack of deposition in lymphoid tissue. The remarkable similarities between Nor98 and the discordant scrapie cases following transmission suggest that the TSE agents responsible for disease represent either a single strain or two closely related strains. Alternatively, Nor98 may represent a sporadic prion disease, albeit one not exactly akin to sCJD [52]. The short protease-resistant fragments seen in Nor98 seem more reminiscent, if anything, of certain forms of the human genetic prion disease GSS [58,59], although N-terminal sequencing of these fragments is awaited to validate or refute this mooted relationship.

#### CWD in deer and elk.

CWD is no newcomer, being recognized as far back as 1967 as a clinical syndrome of unknown etiology. The histopathological and biochemical characteristics have been described in detail [60] and fall within the mainstream of prion diseases. These are illustrated in Figure 2. However, CWD possesses two striking features that warrant our attention. First, it is the only prion disease known to affect free-ranging mule deer, white-tailed deer, and Rocky mountain elk. Second, it is a disease where horizontal spread is readily recognizable [61,62]. With the possible exception of natural scrapie, this stands in contrast to other important prion diseases where horizontal transmission happens by virtue of human activity (e.g., by iatrogenic procedures or industrial cannibalism [63–65]). Likely related to the second point, CWD can attain spectacular “attack rates” in affected populations (approximately 30% in some local populations of deer and essentially 100% in captive research facilities [60]), and is undergoing a swift geographical spread across North America. It is in the context of its almost wildfire spread that CWD is considered an emergent threat (Figure 4). Insofar as moose can be affected (http://www.cwd-info.org), the prospects for colonization of new species in the tundra and boreal forest are truly worrying.

Some aspects of CWD epidemiology are puzzling. As noted, there are two types of affected populations, corresponding to feral and farmed cervids. Insofar as incidences in the two types of populations are both on the rise, they are referred to as epidemics. In the case of free-ranging cervids, an epicenter is located in the contiguous parts of the northeast corner of Colorado, southeast Wyoming, and the extreme southwest corner of Nebraska. Additional cases have been reported in other Rocky Mountain and Great Plains states, as well as more surprising instances in noncontiguous states such as Illinois and Wisconsin (Figure 4). For farmed cervids, instances have been reported in Colorado, Kansas, Oklahoma, Minnesota, Nebraska, South Dakota, Wisconsin, and Wyoming. Appearance in two populations is also the case in Canada (albeit in smaller numbers), where there are four foci of free-ranging animals in the province of Saskatchewan and one focus in Alberta, and incidences in farmed animals in both provinces. Geographic dispersion in farmed animals is attributed to sale and transport of affected individuals, and predicting the future spread of CWD within the captive cervid industry is problematic, as movements are commercially based and unregulated in many states and provinces.

In any event, given the comparative ease with which horizontal spread can be observed in an experimental setting, a causal connection can be posited between the two types of epidemics, e.g., free-ranging infected animals came into contact with farmed animals, or vice versa. However, disparities in geographic distribution have suggested this simple explanation is inadequate [66]. Either the historic origin of a putative point source goes back farther than suggested by current records (with dispersion via migration or cryptic vectors in the years prior to the first recognition of the disease), or, there are CWD epidemics with etiologically distinct origins. For example, isolated pockets of disease may reflect the de novo emergence of sporadic CWD. Given the precedent of BSE, an origin from contaminated feed has to be considered in the case of CWD in farmed cervids. In this instance though the husbandry of these animals does not normally encompass protein concentrate feed additives, and the prion strain of CWD is distinct from BSE (itself rare in North America), making this mechanism of disease spread unlikely.

Perhaps the greatest enigma in the case of CWD is how the disease can spread horizontally. There are reported and anecdotal instances where introduction of one affected animal led to disease in several other members of a farmed herd [67]. Also, physical proximity by penning is claimed to increase disease incidence. An oral route of exposure is inferred from the presence of infectivity in lymphoid tissue of the alimentary canal [68,69], yet the problem remains as to which bodily fluid or secretion contains infectivity. Feces and saliva are posited as being prion-contaminated, but a sighting by way of a prion bioassay has yet to be made. Clearly, definitive knowledge on this point is required for rational control measures, yet there is a partial sense of déjà vu here for earlier failures to identify the mechanism of spread in the “other” prion disease with putative horizontal spread, namely natural scrapie of sheep and goats. Recent work has illustrated the novel idea that chronic inflammation can modify the organ tropism of prions [70], and that infectivity can be detected in the urine of mice with chronic inflammatory kidney disease [71] (albeit assayed by the “sensitive” route of intracerebral inoculation rather than by an oral route that may be more pertinent in vivo). Furthermore, deposits of PrP^Sc^ have been found in the mammary glands of sheep with coincident scrapie infection and mastitis [72]. These results have led to the suggestion that inflammation may play a role in the horizontal spread of prions.

#### Unclassified prion disease in cattle.

Last but not least, large-scale surveillance programs enacted within the European Union and Japan have unearthed several atypical, “waste-basket” prion diseases of cattle with distinct biochemical signatures from BSE. Three cases were identified in France in which an atypical molecular signature was observed (increased size of unglycosylated PrP^res^ and less preponderance for di-glycosylated PrP^res^) [73]. In addition, one abnormal case was identified in Japan with a similar decreased percentage of di-glycosylated PrP^res^, but with a faster mobility of the unglycosylated form [74]. The origins of such cases are enigmatic, with suggestions including infection of cattle with scrapie prions, strain evolution of BSE, or the occurrence of sporadic prion disease in these animals [73].

#### More stars or better telescopes?

Our ability to detect prion diseases is superior to ten years ago, and part of the expansion in the universe of prion diseases is undoubtedly due to large-scale animal screening programs initiated in the wake of BSE. Highly organized human CJD surveillance systems have also made their mark. For CWD, a case can be made that the disease is expanding in the simple sense of the number of affected animals increasing with each passing year. Is this the whole story though? Beyond incidence of cases, is the pan-global diversity of disease types increasing on a yearly basis too? For Nor98, if we are lucky, “look-backs” from archival samples may help us to understand if this new disease is an impostor (i.e., in existence prior to the 1990s). More generally though, the prion hypothesis predicts de novo biogenesis could take place spontaneously. It is possible that insights into the larger question of continuously emerging foci of disease may come first from laboratory rather than from epidemiological studies.

## Deciphering Sporadic Prion Disease

### 

As noted previously, prion diseases are unique within the field of microbiology in having a tripartite (i.e., infectious, genetic, or sporadic) epidemiological manifestation. Perhaps the closest that conventional viruses can approximate this state of affairs would be in the case of retroviruses, where an RNA genome is reverse-transcribed into a cDNA copy. Here, vertical transmission of an infectious state can occur via chromosomal integration of the cDNA copy (provirus) into cells of the germ-line, with subsequent expression of the provirus in somatic cells leading to production of infectious virions. Nonetheless, a functional proviral genome can only appear from a precursor. Thus proviruses cannot appear “out of nowhere,” and retroviruses cannot recapitulate a sporadic epidemiology. In contrast, sporadic epidemiology can be seen as a defining hallmark of prion diseases as transmissible protein folding disorders. However, before probing deeper into this enigmatic epidemiological manifestation, it is worth considering an alternative attribution.

The possibility that some cases of classical sporadic CJD might be caused by an infectious etiology (from BSE, or even BASE-affected animals) begs the larger question as to whether all sporadic prion disease can be accounted for in this fashion, i.e., are attributable to infection by pre-existing prions. This theory has a seeming advantage in its economy, but is it tenable? In the case of natural prion diseases of animals, close scrutiny and clinical assessment of large herds of livestock is difficult to achieve. On the other hand, epidemiological surveillance and neurological scrutiny are performed to higher levels in a medical setting, and so it is to the human population we must turn to best address this issue. Here the sporadic diseases comprise sCJD and sFI, with the bulk of information being available for the former. For the case of BSE as a causative factor, insofar as sCJD (i) predates BSE by decades, (ii) occurs in industrialized countries geographically removed from the UK, and (iii) occurs in people who have never visited the UK; an origin for mainstream sCJD from BSE prions can be absolutely excluded. This leads back to earlier musings on the origin of sCJD [75] where attempts were made to link the disease to the animal reservoirs of disease known at the time, principally scrapie in sheep. These studies were negative. More recent analyses of sCJD epidemiology again stress the role of multiple point source events [76]. From the perspective of an infectious etiology, this requires one to invoke another hypothetical prion disease agent—one that must be widespread to account for the occurrence of sCJD in all countries at a remarkably similar rate. We now know about BASE and Nor98, but to ascribe them this property would be more than premature. In the case of BASE it is not known if this disease is even transmissible. Nor98, though definitely a disease to watch, has a 12-kDa PrP^res^ signature that is (at least in sheep) quite different from that seen in sCJD, making a causal link unlikely. Therefore, in the absence of a widely disseminated reservoir of human-tropic prions that may serve to initiate infections, other mechanisms must be entertained for the origin of sCJD.

The pre-existing infectivity hypothesis (for want of a better label) also runs into problems when one considers animal prion diseases. As we have seen, these may be perpetuated by horizontal spread, but there is a conundrum with regard to origin. Many labs study experimental scrapie in rodents, and these prion isolates are derived from exposure to material from scrapie-infected sheep, but from whence did sheep themselves acquire disease? When did the first scrapied sheep fall from physiological grace to succumb to this neurological disease? (Historical records make it seem quite likely this disease goes back to the 1700s in Europe, and it has been suggested based upon composition of Chinese characters that scrapie existed in Ancient China [77]). A similar question pertains to the first cases of BSE. Were these spontaneous or (leading back to the same question) attributable to a variant form of scrapie in the large UK sheep population? Thus, even if we put aside the other problems, the pre-existing infectivity hypothesis ultimately has to invoke a first spontaneous de novo synthetic event. While impossible in the realm of virology, because we know the prion precursor protein (i.e., PrP^C^) is host-encoded, this type of event does not pose an impasse for the prion hypothesis: it is more a question of “how?” rather than “if.”

#### The prion universe: Big Bang or repeated “singularities”?

Spontaneous prion creation might have happened only once in the Earth's biosphere, a prion Big Bang, so to speak, with all current prion isolates representing the diaspora of this proto-prion. However, there are hints that de novo synthesis events may have happened more than once. Instead of a Big Bang, a perhaps better astrophysical analogy would be the continuous birthing of different varieties of stars from condensation of gas clouds.

The evidence that prions might “ignite” spontaneously—that sporadic disease represents de novo prion synthesis at dispersed points in space and time—is accruing slowly, and is along the following lines. From an epidemiological point of view, excluding the trivial case of spreading CWD in farmed animals by trucking, prion diseases are scattered geographically, and there is no evidence for a universally dispersed yet cryptic prion disease able to cause sCJD on all inhabited continents. sCJD itself has several subtypes and may in turn be different from sFI, again incompatible with a universal sporadic agent and perhaps suggestive of a more stochastic process of biogenesis. Last, there are three types of experiments where infectious prions were created in the lab. In one case this was addressed by overexpression of a *P101L* mutant PrP, followed by transmission to TgP101L (but asymptomatic) indicator mice [78,79]. (Absence of spontaneous disease in low-expresser mice bearing the *P101L* mutation has been noted by several labs, see also [80,81]). In the second case, there was production via inoculation of TgP101L indicator mice with β-sheet conformation synthetic peptides [82], and in the third case by deliberate misfolding of pure recombinant PrP [83]. The experiment with recombinant protein was artificial in that truncated misfolded PrP was inoculated into transgenic mice overexpressing a similarly truncated form of PrP^C^, and the “specific infectivities” (ID_50_ units per mg of total protein) may lie orders of magnitude below those of natural prions. Nonetheless, a precedent may have been established. Just how this all might happen in vivo is not clear, and some possibilities are presented in Table 3. What is also growing clearer, however, is that the “gap” between the properties of cellular prion proteins and their prionized counterparts may be narrower than once believed. Yeast have true-breeding cytoplasmic traits due to protein misfolding (commonly referred to as yeast prions), and there is a debate as to whether the prionized version of the yeast host proteins serve a physiological purpose [84–86]. In the sea-slug *Aplysia,* prion-like states of the neuronal mRNA translation factor CPEB have been posited as stable guardians of synaptic memory [87]. PrP^C^ itself was once thought to be a confirmed singleton, a monomer adhering to an α-helical lifestyle, but it is now known that Cu(II) binding induces conformational changes [88,89] and that N-terminal PrP sequences modulate oligomerization [90], so it is not an enormous stretch to consider whether a version of PrP^C^ capable of templated propagation/perpetuation of a β-sheet state might be present in healthy individuals. In vitro, PrP^C^ is capable of refolding to quasi-PrP^Sc^-like, albeit non-infectious β-oligomeric forms using chemical denaturation and acidification [9,91], while thermal denaturation and manipulation of detergent conditions can lead to formation of PrP27–30 [92]. Further work to explore the boundaries of PrP^C^'s behaviour and ways to subvert this molecule in vitro (e.g., facilitate these conformational transitions under kinder, gentler conditions) is eagerly awaited.

**Table 3:** Hypothetical Mechanisms for De Novo Creation of Prion Infectivity

## Conclusion

While some recent prion crises may be man-made (amplification of BSE), and some emerging diseases may be exacerbated by human actions (trucking of CWD-affected deer), it is extremely unlikely that the origins of *all* emerging prion disease can be blamed on Homo sapiens. Tackling the larger questions—and enigmas—of prion biology will be important if we are to deal with emerging prion diseases in a pro-active rather than a reactive manner. Horizontal spread may either occur directly between infected animals or involve the intervention of an environmental reservoir, but to be brought under control these processes will need to be demystified and defined in terms of explicit biochemical entities. Sporadic prion diseases may emerge continuously from molecular wear and tear of PrP^C^ (an abundant neuronal protein), and we need to understand the ins and outs of this process, too. Cell biological systems or transgenic systems to gently abuse PrP^C^ are urgently needed to supplant the harsh conditions currently used in vitro. New diagnostics should be brought to bear upon questions raised by emergent diseases, and here PMCA may be particularly adept because of sensitivity and because the process may be modified to be informative about in vivo replicative mechanisms.

Where will the next prion epidemics emerge? During the height of the BSE epidemic, meat and bone meal was exported from the UK to non-European countries, and the sequelae of these actions may yet to be felt. If in vivo systems for de novo biogenesis can be made robust, an inevitable conclusion is that sporadic prion diseases can appear anywhere on the planet where there are large populations of livestock. As yet unscathed, continents in the Southern hemisphere may be home for the epidemics of the 21st century. Fortunately, in dealing with the problems of emergent syndromes we may note that sporadic disease has one shining virtue—it is extremely rare, with an incidence of between one and two cases per 2 million head of population. While we put great faith in human ingenuity to tease apart the processes of prion replication, dissemination, and biogenesis, this biological obstacle may be a crucial ally in keeping the prion expansion within reasonable bounds.

## Supporting Information

### Accession Numbers

PrP protein sequences from SwissProt (http://www.ebi.ac.uk/swissprot) are cattle (PRIO1_BOVIN), elk (PRIO_CEREN), human (PRIO_HUMAN), mouse (PRIO_MOUSE), mule deer (PRIO_ODOHE), and sheep (PRIO_SHEEP). *PRNP* gene sequences from Entrez GeneID (http://www.ncbi.nlm.nih.gov/entrez) are cattle *Prnp* (281427), human *PRNP* (5621), mouse *Prnp* (19122), and sheep *Prnp* (493887).

## Abbreviations

BASE: bovine amyloidotic spongiform encelphalopathy
BSE: “mad cow” disease
CJD: Creutzfeldt-Jakob disease
CWD: chronic wasting disease
PMCA: protein misfolding cyclic amplification
PrP: prion protein
sCJD: sporadic Creutzfeldt-Jakob disease
sFI: sporadic fatal insomnia
TSE: transmissible spongiform encephalopathies
vCJD: variant Creutzfeldt-Jakob disease
